# Analysis of Clinical Characteristics of 52 Patients with Uveitis before and after Vitrectomy and Factors Affecting Clinical Efficacy

This article has been retracted.

**DOI:** 10.1155/2021/4000531

**Published:** 2021-10-27

**Authors:** Qian Liu, Yinghong Zhou, Hongxia Deng, Xiaoxia Xiang, Chaohua Chen, Chao Wang, Ran Huang

**Affiliations:** ^1^Department of Ophthalmology, Chongqing Fengdu People's Hospital, Chongqing 408200, China; ^2^Department of Ophthalmology, Zaozhuang Municipal Hospital, Zaozhuang, Shandong 277102, China

## Abstract

**Objective:**

To investigate the pre- and postsurgical clinical characteristics and clinical efficacy of patients with uveitis.

**Methods:**

The clinical data of patients with uveitis who underwent vitrectomy in our hospital from March 2019 to February 2021 were retrospectively analyzed. There were 52 cases of 64 eyes in total. The data on patient's gender, age, etiology, course of disease, anatomical classification, number of recurrences, changes in vision before and after surgery, changes in eye signs before and after surgery, and occurrence of postoperative complications were collected. The clinical features before and after vitrectomy were compared, and the influencing factors of clinical efficacy were analyzed.

**Results:**

The ocular signs of patients with uveitis after vitrectomy were significantly improved compared with before operation, and the difference was statistically significant (*P* < 0.05). The visual acuity after vitrectomy in patients with uveitis was significantly improved compared with that before operation, and the difference was statistically significant (*P* < 0.05). There was no significant difference in the surgical treatment of uveitis patients of different gender, age, and etiology (*P* > 0.05). There are significant differences in the clinical efficacy of vitrectomy in patients with different anatomical classifications. Among them, patients with panuveitis have the best clinical efficacy with vitrectomy and patients with posterior uveitis have the worst clinical efficacy with vitrectomy (*P* < 0.05). There is a significant difference in the clinical efficacy of vitrectomy in patients with recurrence times. The lower the number of recurrences, the better the clinical efficacy of vitrectomy in patients (*P* < 0.05).

**Conclusion:**

There are significant differences in the clinical signs of patients with uveitis before and after vitrectomy. Vitrectomy is effective in the treatment of uveitis. The type of anatomy and the number of recurrences are influencing factors for the clinical efficacy of vitrectomy. For patients with posterior uveitis, the surgical method should be carefully considered or a more reasonable treatment method should be selected, and for patients with uveitis with less recurrence, vitrectomy should be considered for active treatment.

## 1. Introduction

Uveitis is a common disease in ophthalmology, with redness, eye pain, and decreased vision as the main clinical symptoms, with eye congestion, aqueous humor opacity or oozing, vitreous inflammatory opacity, retinal edema, hemorrhage, and so on as the main signs. The disease has a high incidence in young adults. It is easy to recur, and treatment is difficult. If treatment is delayed or improperly handled, it can cause blindness in patients [1]. Therefore, the relevant research on uveitis has been valued by ophthalmologists all over the world. The most effective treatment at this stage is the use of immunosuppressive agents, which can achieve certain effects, but long-term treatment will produce side effects, which can cause immune disorders in severe cases and seriously affect the physical and mental health of patients [2, 3]. In addition, uveitis can also cause a variety of serious complications such as vitreous opacity or hemorrhage, vitreoretinopathy, and retinal detachment. The above complications cannot be treated with drugs and require surgical treatment, such as vitreous surgery and laser photocoagulation. Studies have shown that the prognosis of patients with uveitis undergoing vitrectomy has been improved to some extent [4], but there are still some patients with poor surgical results and poor postoperative prognosis. Therefore, the author believes that it is necessary to actively explore the clinical features before and after vitrectomy and the influencing factors of clinical efficacy. This study retrospectively analyzed the clinical characteristics of 52 patients with uveitis before and after vitrectomy and at the same time discussed the factors affecting the clinical efficacy. It is intended to provide guidance for clinical selection of the correct treatment method, improvement of surgical efficacy, and improvement of patient prognosis. The report is as follows.

## 2. Research Objects and Methods

### 2.1. Research Object

This study included patients with uveitis who underwent vitrectomy in our hospital from March 2019 to February 2021, with a total of 52 cases and 64 eyes. All patients met the diagnostic criteria for uveitis in the “Uveitis Diagnosis and Treatment” [5], and the following patients were excluded: (1) patients with other infectious eye diseases, patients with glaucoma-cyclitis syndrome; (2) medications not prescribed by the doctor, the treatment is not standardized, and the medication is stopped halfway through the poor compliance; (3) the patients with mental illness and other malignant tumors; (4) the patients with severe heart, liver, kidney, and other organ diseases; and (5) the information is incomplete. All vitrectomy procedures are performed by the same medical team in our hospital.

### 2.2. Data Collection

The patient's gender, age, etiology, course of disease, anatomical classification, number of recurrences, changes in vision before and after surgery, changes in eye signs before and after surgery, and occurrence of postoperative complications were collected. Among them, the visual acuity and ocular signs before and after the operation were routinely checked upon admission and discharge. The intraocular pressure was measured with a noncontact tonometer, the anterior segment was examined with a slit lamp microscope, and the fundus was examined with a direct ophthalmoscope. Binocular indirect ophthalmoscope, front lens, and three-sided mirror are used for detailed inspection, and the patient's vision, conjunctiva, cornea, anterior chamber, iris, pupil, lens, vitreous, retina, and intraocular pressure are recorded in detail during admission and discharge.

### 2.3. Judgment of Clinical Efficacy [6–8]

(1) Cured: the patient's conscious symptoms disappeared, the visual acuity or corrected visual acuity reached 1.0 or above, no corneal edema, posterior corneal KP (-), anterior chamber inflammatory cells (-), aqueous humor (-), pupil drug-induced fully enlarged, no posterior iris adhesions, and normal eyes. (2) Significantly effective: the patient's eye symptoms are significantly improved, visual acuity or corrected visual acuity is improved by ≥4 lines (one line for every 0.02 between 0.01 and 0.1), corneal edema is significantly relieved, corneal KP is significantly reduced, and anterior chamber inflammatory cells are significantly reduced. The flashing of aqueous humor was significantly weakened, the anterior chamber empyema basically disappeared, the pupils were dilated with drugs, no posterior iris adhesions were seen, and the optic papilla and macular edema of the fundus subsided. (3) Effective: the patient's eye symptoms have improved, visual acuity or corrected visual acuity has improved by ≥2 lines, corneal edema has been relieved, corneal KP has been reduced, anterior chamber inflammatory cells have been reduced, aqueous humor has been reduced, and iris has been mild or moderate. After the degree of adhesion, the optic papilla and macular edema of the fundus were alleviated. (4) Invalid: the patient's eye symptoms have no obvious changes or even worsened, visual acuity has not been significantly improved or even decreased, corneal edema is still present, corneal KP has not decreased, anterior chamber inflammatory cells have not decreased or even increased, aqueous humor flashing has not changed, and iris has been moderate or severe postadhesion, but still see fundus optic papilla and macular edema.

### 2.4. Standards for Grading and Quantifying Eye Signs

The grading and quantification of ocular signs in patients with uveitis are evaluated according to the standards established in the literature [8], as shown in Table 1.

### 2.5. Statistical Methods

SPSS 22.0 statistical software was used to process and analyze the data of this study. Measurement data are expressed by ($\bar{x}$ ± *s*) using the *t* test; count data are described by frequency or percentage using the *χ*2 or rank-sum test. The difference was statistically significant when *P* < 0.05.

## 3. Result

### 3.1. General Condition of the Patients

In this study, 52 patients with uveitis had 64 diseased eyes, including 40 males with 48 eyes and 12 females with 16 eyes. Age of onset: 8 cases (15.38%), ≤20 years old; 28 cases (53.85%), 21–40 years old; 10 cases (19.23%), 41–60 years old; and 6 cases (11.54%), ≥61 years old. Causes of disease: 29 cases (55.77%) of idiopathic uveitis, 7 cases (13.46%) of traumatic uveitis, 4 cases (7.69%) of ankylosing spondylitis combined with uveitis, uveitis after intraocular lens operation in 3 cases (5.77%), rheumatoid arthritis with uveitis in 3 cases (5.77%), Vogt–Koyanagi–Harada syndrome in 3 cases (5.77%), and tuberculosis with uveitis in 3 cases (5.77%). Anatomical classification: 38 eyes (59.38%) with anterior uveitis, 3 eyes (4.69%) with intermediate uveitis, 5 eyes (7.81%) with posterior uveitis, and 18 eyes (28.13%) with panuveitis. Clinical efficacy: 4 eyes were cured (6.25%), 20 eyes were markedly effective (31.25%), 32 cases were effective (50.0%), and 8 eyes were ineffective (12.50%).

### 3.2. Changes of Eye Signs before and after Vitrectomy in Patients with Uveitis

The ocular signs of patients with uveitis after vitrectomy were significantly improved compared with before operation, and the difference was statistically significant (*P* < 0.05), as shown in Table 2.

### 3.3. Comparison of Visual Acuity before and after Vitrectomy in Patients with Uveitis

The visual acuity after vitrectomy in patients with uveitis was significantly improved compared with that before operation, and the difference was statistically significant (*P* < 0.05), as shown in Table 3.

### 3.4. Analysis of Factors Affecting the Clinical Efficacy of Vitrectomy in Patients with Uveitis

#### 3.4.1. The Influence of Gender on the Clinical Efficacy of Vitrectomy

There was no statistically significant difference in the clinical efficacy of vitrectomy in patients of different genders (*P* > 0.05), as shown in Table 4.

#### 3.4.2. The Influence of Age on the Clinical Efficacy of Vitrectomy

There was no statistically significant difference in the clinical efficacy of vitrectomy in patients of different ages (*P* > 0.05), as shown in Table 5.

#### 3.4.3. The Influence of Etiology on the Clinical Efficacy of Vitrectomy

There was no statistically significant difference in the clinical efficacy of vitrectomy in patients with different etiologies (*P* > 0.05), as shown in Table 6.

#### 3.4.4. The Influence of Anatomical Classification on the Clinical Efficacy of Vitrectomy

There are significant differences in the clinical efficacy of vitrectomy in patients with different anatomical categories. Among them, patients with panuveitis have the best clinical efficacy of vitrectomy and patients with posterior uveitis have the worst clinical efficacy of vitrectomy. The difference is statistically significant (*P* < 0.05), as shown in Table 7.

#### 3.4.5. The Influence of the Number of Recurrences on the Clinical Efficacy of Vitrectomy

There are significant differences in the clinical efficacy of vitrectomy in patients with different recurrence times. The lower the recurrence times, the better the clinical efficacy of vitrectomy in patients, and the difference is statistically significant (*P* < 0.05), as shown in Table 8.

## 4. Discussion

### 4.1. Clinical Characteristics of Patients with Uveitis

The results of this study showed that the proportion of male uveitis patients was significantly higher than that of females (3.33 : 1), which was consistent with the domestic research results of Zhang et al. [9] and Li et al. [10], indicating that uveitis was more common in our country male, but some foreign reports [11, 12] show “female than male,” the reason might be that there were regional differences in the incidence of the disease. In this study, the age of onset was mostly 21–40 years, suggesting that uveitis occurs frequently in young adults, which was consistent with reports at home and abroad [13–15]. Common causes of uveitis were idiopathic uveitis, traumatic uveitis, ankylosing spondylitis with uveitis, uveitis after intraocular lens surgery, rheumatoid arthritis with uveitis, Vogt–Koyanagi–Harada syndrome, and tuberculosis combined with uveitis. In this study, 29 cases were mainly idiopathic uveitis, accounting for 55.77%, followed by 7 cases (13.46%) of traumatic uveitis and 4 cases of ankylosing spondylitis combined with grapevine meningitis (7.69%), which was consistent with previous reports at home and abroad [13–15].

The anatomical location can reflect the area affected by inflammation. In this study, anterior uveitis had the highest proportion, followed by panuveitis and then posterior uveitis and intermediate uveitis, which was similar to previous reports [16, 17]. Anterior uveitis includes iritis, anterior cyclitis, and iridocyclitis. Studies have suggested that the pathogenesis of panuveitis might be related to the activation of receptors of the innate immune system to cause G-bacterial infection, and the ocular tissue damage caused by acute anterior uveitis will promote the release of endogenous inflammatory factors and maintain and aggravate inflammation in the eye. Patients with acute anterior uveitis usually present with redness, eye pain, photophobia, and tearing. In intermediate uveitis, the inflammatory factors mainly accumulate in the vitreous, and its pathogenesis is still unclear. The patient's onset was insidious and relatively slow. It was often not accompanied by symptoms such as jealous, eye pain, photophobia, and tearing and no obvious clinical symptoms. Such patients were often mildly ill, but there were also a few cases of vitreous hemorrhage, leading to a sudden drop in vision. Posterior uveitis was caused by inflammatory factors that affect the blood vessels of the choroid, retina, and optic nerve head. Choroiditis, retinitis, and retinal vasculitis are common. The symptoms of these patients were related to the affected site and inflammation. Panuveitis referred to a mixed type of multiple types of uveitis. Panuveitis includes not only inflammation of the entire uvea but also inflammation of the retina and vitreous. Studies have shown that as patients age, the incidence of panuveitis will decrease [18].

### 4.2. Vitrectomy in Patients with Uveitis and Its Clinical Efficacy Analysis

Vitrectomy has a clear curative effect in the treatment of uveitis. The main mechanism of the operation is to clear specific antigens in the vitreous, remove nonspecific inflammatory factors, self-assisting cells, and chemokines that accumulate in the vitreous, and remove toxic substances, inflammatory factors, and lesions. At the same time, the vitreous body can be injected into the eye through the surgical incision, which provides a way for the treatment of fundus lesions and can further clarify the cause of uveitis [19, 20]. The results of this study showed that there were significant differences in visual acuity and eye signs in 52 patients with uveitis before and after vitrectomy, indicating that vitrectomy is effective in treating uveitis.

This study further analyzed the differences in the therapeutic effects of vitrectomy for uveitis patients of different ages, genders, etiology, anatomical classifications, and recurrence times. The results showed that the surgical treatment effects of uveitis patients of different genders, ages, and etiology were not effective. However, it was found that there were significant differences in the clinical efficacy of vitrectomy in patients with different anatomical classifications. Among them, patients with panuveitis had the best clinical efficacy of vitrectomy and patients with posterior uveitis had the worst clinical efficacy of vitrectomy. In patients with different recurrence times, there is a significant difference in the clinical efficacy of vitrectomy. Among them, the fewer the relapses, the better the clinical efficacy of vitrectomy. This suggests that the clinical efficacy of vitrectomy in patients with posterior uveitis is poor, while the lower the number of recurrences of uveitis, the better the clinical efficacy. Therefore, for patients with posterior uveitis, we should carefully consider the operation method or choose a more reasonable treatment method. For patients with less recurrent uveitis, vitrectomy should be considered for active treatment.

In summary, there are significant differences in the clinical signs of patients with uveitis before and after vitrectomy. Vitrectomy is effective in treating uveitis. The type of anatomy and the number of recurrences are factors that affect the clinical efficacy of vitrectomy. For patients with uveitis, we should carefully consider vitrectomy or choose a more reasonable treatment method, and for patients with uveitis with fewer recurrences, vitrectomy should be considered for active treatment.

## Figures and Tables

**Table 1:** Grading and quantification standards for eye signs.

Grading of eye signs	Conjunctiva	Cornea	Anterior chamber	Iris	Pupil	Fundus
Normal	Normal	Normal	Normal	Normal	Normal or drug-induced full dispersal	Normal
Mild	Conjunctival hyperemia	Edema, KP (+)	Flash of water (+)–(++) Inflammatory cells (+)–(++)	Dark color	Shrink, less than or equal to 1/3 of the iris after adhesion	Edema around the retina, no bleeding or exudation
Moderate	Ciliary hyperemia	Edema, KP (++)	Flash of water (+++)–(++++) Inflammatory cells (+++)–(++++)	Dark color, unclear texture	Shrink, 1/3–2/3 behind iris adhesion	Bleeding, oozing
Severe	Mixed hyperemia	Edema, KP (+++)	Empyema and exudation	Cannot see clearly	More than 2/3 of posterior iris adhesion, see exudate membrane	Retinal detachment or macular edema, papilledema or unclear vision

**Table 2:** Visual changes before and after vitrectomy in patients with uveitis (*n* = 64).

Eye signs	Preoperative				Postoperative				Z	*P*
	Normal	Mild	Moderate	Severe	Normal	Mild	Moderate	Severe		
Conjunctiva	5	7	15	37	26	28	10	0	7.644	<0.001
Cornea	7	11	42	4	59	4	1	0	9.204	<0.001
Anterior chamber	6	39	15	4	57	6	1	0	8.715	<0.001
Iris	7	29	25	3	52	11	1	0	8.109	<0.001
Pupil	10	27	14	13	51	11	2	0	7.422	<0.001
Fundus	38	6	4	16	55	3	3	3	3.495	<0.001

**Table 3:** Comparison of visual acuity before and after vitrectomy in patients with uveitis (*n* = 64).

Time	No light-sensitive	Light-sensitive	Manual	Vision index	0.01–<0.1	0.1–<0.3	0.3–<0.6	0.6–<1.0	≥1.0
Preoperative	3	13	8	8	16	10	5	1	0
Postoperative	1	4	2	3	10	18	16	9	1
Z	5.184								
*P*	<0.001								

**Table 4:** Comparison of clinical efficacy of vitrectomy in patients of different genders (*n* = 64).

Gender	Eye count	Cured	Markedly effective	Efficient	Invalid
Male	48	2	16	24	6
Female	16	2	4	8	2
Z		0.2303			
*P*		0.839			

**Table 5:** Comparison of clinical efficacy of vitrectomy in patients of different ages (*n* = 64).

Age	Eye count	Cured	Markedly effective	Efficient	Invalid
≤20 years	10	1	2	6	1
21–40 years	33	2	10	18	3
41–60 years	13	1	6	5	1
≥61 years	8	0	2	3	3
H		3.558			
*P*		0.131			

**Table 6:** Comparison of clinical efficacy of vitrectomy in patients with different etiologies (*n* = 64).

Cause	Eye count	Cured	Markedly effective	Efficient	Invalid
Idiopathic	30	2	8	17	3
Traumatic	9	0	3	4	2
Ankylosing spondylitis	5	0	2	2	1
After intraocular lens surgery	5	1	1	2	1
Rheumatoid arthritis	4	1	1	2	0
Vogt–Koyanagi–Harada syndrome	6	0	3	3	0
Tuberculosis	5	0	2	2	1
H		1.958			
*P*		0.924			

**Table 7:** Comparison of clinical efficacy of vitrectomy in patients with different anatomical classifications (*n* = 64).

Anatomical type	Eye count	Cured	Markedly effective	Efficient	Invalid
Anterior uveitis	38	1	11	23	3
Intermediate uveitis	3	0	1	1	1
Posterior uveitis	5	0	0	2	3
Panuveitis	18	3	8	6	1
H		121.110			
*P*		0.007			

**Table 8:** Comparison of clinical efficacy of vitrectomy in patients with different recurrence times (*n* = 64).

Number of relapses	Eye count	Cured	Markedly effective	Efficient	Invalid
≤2	45	4	16	23	2
3–4	12	0	4	6	2
≥5	7	0	0	3	4
H		11.487			
*P*		0.003			

## Data Availability

The data used during the current study are available from the corresponding author.
